# Nursing Method of Patients with Severe Traumatic Brain Injury and Fracture in the Ambulance

This article has been retracted.

**DOI:** 10.1155/2022/2652916

**Published:** 2022-09-07

**Authors:** Haihua Zhang, Min Zhang, Fengqing Zhao

**Affiliations:** ^1^Emergency Department, Yantai Yuhuangding Hospital, Yantai, 264000 Shandong, China; ^2^Intensive Care Unit of Neurology, Yantai Yuhuangding Hospital, Yantai, 264000 Shandong, China

## Abstract

Craniocerebral injury accounts for 9%-21% of the injuries in all parts of the body, and the incidence rate ranks first in all types of trauma or only lower than limb fractures. This study mainly discusses the nursing methods of patients with severe traumatic brain injury and fractures in ambulances. This study is based on risk factors with moderate-to-higher association strength from retrospective studies. According to the regression coefficients of the logistic regression model, the risk factors were assigned, and the early warning score table of craniocerebral injury complicated with hyponatremia was established. The energy efficiency of the early warning score table was evaluated by case diagnostic test and ROC analysis. At the same time, risk grading is carried out, and the chi-square test is used to test the reliability of the grading standard, so as to identify the risk of hyponatremia in patients with craniocerebral injury early and screen out high-risk patients as the key observation objects of nurses. Based on the early warning score table of craniocerebral injury complicated with hyponatremia, different systematic nursing intervention measures were taken for low-risk patients and high-risk patients, and their application effects were evaluated. The clinical application effect of the systematic nursing intervention program was evaluated by the historical control research method, which provided a reference for the nursing in the ambulance to prevent other complications of patients with craniocerebral injury. The positive rate of prehospital operation can reach 64.44%, and the specific rate can reach 84.44%. 60% of the sample sought better metastatic care in terms of the purpose of using an ambulance. The systematic nursing intervention program has a certain effect on reducing the incidence of hyponatremia in patients with craniocerebral injury and shortening the hospitalization time of patients with craniocerebral injury. The early warning score of craniocerebral injury complicated with hyponatremia developed in this study is concise and practical and can provide a basis for clinical assessment of the risk of hyponatremia in patients with craniocerebral injury.

## 1. Introduction

Managers should pay attention to the accident knowledge education of nurses with different characteristics. Better knowledge of prehospital emergency care can make care in the ambulance easier and reduce the infection rate of patients. For nurses with advanced age, high education, and high professional titles, they should improve their accident knowledge training to maintain the accident knowledge level of the whole nursing team. At the same time, strengthening accident rescue drills and enhancing nurses' accident rescue experience through scenario drills will help improve nurses' accident knowledge. The opportunities of early shifts in departments, nursing rounds, and group teaching should be actively used, promoting the learning of accident knowledge through theoretical lectures, scenario reproduction, and group discussions. As a professional public health institution, emergency centers (stations) are closely related to the lives and health of the people. They are the forefront of rescuing patients and have obvious medical and social benefits. Moreover, the prehospital medical emergency in the region should be adapted to the local, social, and economic development conditions and the needs of emergency services. Therefore, to carry out research on the construction and management of the prehospital medical emergency system is to promote emergency centers (stations) to provide better quality. It is an essential process for prehospital medical emergency services that are more efficient and better suited to the actual needs of the masses.

Nurses have multiple identities as nurses, educators, and psychological supporters in accident rescue, which requires accident training to take into account all aspects of accident rescue, especially psychological rescue skills which refers to providing humanitarian support to those who have suffered trauma and need support. This is related to whether the victims can reintegrate into society and rebuild their confidence in life after the disaster. Therefore, nursing managers should comprehensively plan the content of accident training, combine diversified training methods, and make full use of social and cultural support to meet the mental health needs of nursing rescue team members, by holding emotional and mental health training courses, providing desktop and on-site crisis simulation exercises to promote the improvement of various accident skills of clinical nurses. This research fills the blank of comprehensive and systematic research on prehospital medical emergency and integrates the modules of legislative guarantee, emergency mode, infrastructure construction, resource allocation, and rescue dispatch to build an interconnected and organic prehospital emergency system.

The junior nurses have gradually become the main force of the nursing team, and the number of nurses with a bachelor's degree or below who graduate every year is still relatively large. Therefore, hospital administrators in this region pay special attention to the comprehensive development of low-level nurses' theoretical knowledge, skills, and management ability, which promotes the development of clinical low-level nurses' accident management ability. Nursing managers should increase the opportunities for nurses to participate in accident rescue experience, build an emergency medical service system, expand and strengthen theoretical and skill training, and establish nursing education institutions with formal training qualifications. Develop targeted accident nursing courses and disaster prevention procedures according to the characteristics of nurses, strengthen disaster nursing construction, and organize training regularly to improve nurses' accident knowledge, accident skills, accident management, and overall accident preparedness. The article firstly adopts the factor analysis method for the specific index innovation of the construction and management of the municipal emergency center, grasps the status of prehospital medical emergency construction and management in each city from a macro perspective, and then analyzes the operation status of the emergency center and the maturity of construction management. For nonemergency transportation services, in the factor analysis, the KMO value is 0.801.

## 2. Related Work

The treatment and care of patients with craniocerebral injury during hospitalization not only require the participation of medical staff but also require family members to undertake a large part of the care work. Taylor et al. believe that traumatic brain injury (TBI) has short- and long-term adverse clinical outcomes, including death and disability. TBI can be caused by a number of major mechanisms, including motor vehicle crashes, falls, and assaults. He described the estimated incidence of TBI-related emergency department (ED) visits, hospitalizations, and deaths in 2013 and compared them with similar estimates in 2007. State-based administrative healthcare data were used to calculate estimates of TBI-related ED visits and hospitalizations based on primary mechanism of injury, age group, gender, and injury intent. Categories of intent to harm include unintentional (motor vehicle collision, fall, being struck by or hitting an object, and unspecified mechanism), intentional (self-harm and assault/homicide), and undetermined intent. These health records are derived from the Healthcare Sample and Utilization Project's National Emergency Department Sample and National Inpatient Sample [1]. Arciniegas and Mcallister believe that traumatic brain injury (TBI) results in approximately 230,000 hospitalizations each year in the United States. Advances in acute treatment of TBI have improved survival after TBI. Many TBI survivors develop neurobehavioral disturbances during the acute postinjury phase. Neurobehavioral sequelae present clinical management challenges for critical care professionals. He defines and describes TBI and reviews its common neuroanatomical and neurobehavioral consequences. These disturbances are organized within the framework of posttraumatic encephalopathy, and the characteristic forms and recovery phases of this condition are discussed. He provides advice on the assessment and management of posttraumatic neurobehavioral problems in the intensive care setting [2]. Jassam et al. believe that traumatic brain injury (TBI) is a major cause of morbidity and disability with a considerable socioeconomic burden. The heterogeneity of pathoanatomical subtypes and the diversity of pathogenesis and extent of injury contribute to differences in the course and outcome of TBI. Following a primary injury, extensive and long-lasting injury continues through a complex cascade of events called “secondary injury.” In animal and human studies, neuroinflammation has been recognized as an important actionable aspect of secondary injury. Because neuroinflammation can be detrimental or beneficial, it is necessary to better understand the timing and complexity of immune responses following TBI before developing immunomodulatory therapies. With the rapidly increasing literature, a clear summary of TBI neuroimmunology is needed. This review presents the current understanding of the immune response to TBI in a chronological and compartment-based manner, emphasizing early changes in gene expression and initial signaling pathways leading to activation of innate and adaptive immunity. Based on recent advances in the understanding of innate immune cell activation, he proposed a new paradigm to study innate immune cells after TBI [3]. Liu et al. associate a stromal cell protein tenascin-C with early brain injury after experimental subarachnoid hemorrhage (SAH). He first assessed the role of another stromal cell protein, periostin, and its relationship to tenascin-C in early brain injury after SAH. Wild-type (*n* = 226) and tenascin-C knockout (*n* = 9) C57BL/6 male adult mice underwent sham or filament punch SAH modeling. Vehicle, anti-periostin antibody, or recombinant periostin was administered randomly by intracerebroventricular injection 30 minutes after modeling. Neuroscore, SAH grade, brain water content, immunostaining, and western blot were assessed blinded 24 to 48 hours after SAH. Periostin was induced in brain capillary endothelial cells and neurons 24 hours after SAH. Anti-periostin antibodies ameliorated post-SAH neurobehavior, brain edema, and blood-brain barrier disruption associated with tenascin-C downregulation, p38 inactivation, extracellular signal-related kinase 1/2, and matrix-related [4]. Thelin et al. have introduced protein markers of pathophysiological processes and tissue fate in the clinic in order to improve injury assessment of brain injury. The most studied protein “biomarker” of brain damage in traumatic brain injury (TBI) is the protein S100B. The purpose of his narrative review was to thoroughly analyze the properties and capabilities of this biomarker, with a focus on assessing its clinical utility in patients with TBI. S100B has been successfully implemented in the clinical area, to screen patients with mild TBI, to assess the need for computed tomography of the head, to predict outcomes in patients with moderate to severe TBI, to detect the development of secondary lesions in patients with brain injury, and to assess treatment effects. The potential opportunities and pitfalls of S100B in different fields usually refer to its specificity and sensitivity in detecting and assessing intracranial injuries [5]. The average anxiety level of family members of craniocerebral injury patients is higher than that of family members of other patients. This may be mainly due to the sudden nature of the traumatic brain injury disease itself. When the patient is first admitted to the hospital, the patient's family is unfamiliar with the hospital layout, the patient's doctor in charge, and the responsible nurse, and the treatment of the disease and the patient's future rehabilitation effect are also uncertain, even faced with the threat of death of loved ones at any time. This can easily make family members extremely worried and panic and lead to a sense of uncertainty about the disease.

## 3. Nursing Methods of Patients with Severe Craniocerebral Injury and Fractures in the Ambulance

### 3.1. Data Sources

1. The selected cases were patients with craniocerebral injury who were discharged from January 2018 to December 2019 in a comprehensive tertiary hospital
2. All the included patients were hospitalized for more than 3 days and were diagnosed with craniocerebral injury, including concussion, skull fracture, and brain herniation, after clinical diagnosis and head CT examination. They did not include cases of isolated scalp injury, chronic subdural hematoma, and skull defect; age ≥ 15 years
3. Patients with abnormal thyroid and adrenal function were excluded; patients with hypernatremia after admission were excluded. A total of 79,480 patients with severe craniocerebral injury and fractures were collected

According to the admission diagnosis, concussion, cerebral contusion, skull fracture, and brain herniation were divided into two groups with and without.

1. According to the surgical method, the patients were divided into three groups: hematoma removal, drilling and drainage, and debridement and suture. Each group was further divided into two groups: with and without
2. According to whether there is coinfection and high fever, they are divided into two groups: yes and no. Infections include pulmonary infection, intracranial infection, and urinary tract infection. Hyperthermia was defined as a body temperature higher than 38 degrees during hospitalization for two or more days
3. The patients were divided into two groups according to whether the patients were fasted or not and whether vomiting occurred
4. According to the past history of hypertension and diabetes, the patients were divided into two groups: with and without

This study mainly explored the effects of systematic nursing interventions on hyponatremia in patients with craniocerebral injury, which belonged to a quasiexperimental study. Therefore, the estimation of the sample size of the experimental study can be taken [6].

(1) $$\begin{array}{c} N=\left(U_{\alpha }+U_{\beta }\right)\cdot \frac{2P\left(1-P\right)}{{\left(P_{1}-P_{2}\right)}^{2}}. \end{array}$$

Condition evaluation function [7, 8]:

(2) $$\begin{array}{c} f\left(x_{1},x_{2},x_{3},\cdots ,x_{n}\right)=\alpha_{1}x_{1}+\alpha_{2}x_{2}+\cdots +\alpha_{n}x_{n}. \end{array}$$

Among them, *α*_1_, *α*_2_, *α*_3_, ⋯, *α*_*n*_ is the weight coefficient, which is the reflection of the contribution to *f* under the same percentage increment.

Assuming that the contribution of each index to the judgment result is the same, a total judgment function is obtained [9]:

(3) $$\begin{array}{c} G=\beta_{1}\left[v\left(f_{1}\right)+\chi \left(f_{2}\right)+\gamma \left(f_{3}\right)+\mu \left(f_{4}\right)\right]. \end{array}$$

Among them,

(4) $$\begin{array}{c} v\left(f\right)=\left\{\begin{array}{cc} 1, & f>0,\\ 0, & f\leq 0, \end{array}\right.\\ f\left(x_{1},x_{2},x_{3}\right)=4x_{1}-3x_{2}-2x_{3}, \end{array}$$

where *x* is the relevant variable.

### 3.2. First-Aid Measures

Due to differences in social and economic development, geographical characteristics, population density, and other factors in different regions, the development of prehospital emergency medical services is not balanced. Each region fully considers its own situation and combines the advantages and disadvantages of different models to carry out local prehospital emergency models. The choice of the national unified prehospital first aid model has not yet been formed.

An analysis database was established, in which variables included call time, reaction time, basic information of patients with severe craniocerebral injury and fractures, cause of injury, injury site, injury address, prehospital index (systolic blood pressure, pulse, respiration, and consciousness), and other research indicators [10].

According to the ability scope of prehospital emergency work after traumatic brain injury, there are requirements of key items of prehospital emergency care for traumatic brain trauma and the characteristics of prehospital emergency treatment of guiding trauma. In this study, the main points of prehospital first aid for craniocerebral trauma were integrated into the trauma information collection table, including pulse oximetry monitoring (it measures the oxygen level in the blood), state of consciousness assessment, and pupil observation. The maintenance of airway patency, resuscitation, and prevention of brain herniation are listed in the prompt section under prehospital diagnosis. At the same time, the medical record information of craniocerebral trauma was edited into 26 medical record identification information of 4 grades (I-IV). Among them, I represents the type of craniocerebral injury, which is a single choice. II-IV represent the characteristic symptoms and signs of traumatic brain injury, divided into common options and unique options. III can make multiple choices, and IV needs to make single choice and fill in. The specific identification information is shown in Table 1.

Open injuries: there are wounds with skin injuries, some of which often bleed, and closed injuries are easy to be misdiagnosed and mistreated. Because open injuries have wound bleeding, more emphasis is usually placed on timely treatment.

Closed injuries: usually there is no wound, and there may be no skin bleeding. Since there is no wound, closed injury combined with visceral injury is usually ignored in the early stage, which can easily lead to misdiagnosis and delayed treatment.

### 3.3. Early Warning Score for Patients with Severe Traumatic Brain Injury and Fractures

The prediction model based on the characteristics of the emergency medical service system can quantitatively reflect the severity and type of traumatic brain injury fractures, but simple indicators cannot accurately reflect the condition and prognosis. The constructed prediction model based on the baseline characteristics of patients in emergency hospital and the characteristics of emergency medical service system and blood biochemical indexes has high prognostic discrimination ability in both the training group and the test group.

- Case Grouping. Patients with craniocerebral injury were divided into hyponatremia group and normal serum sodium group according to whether hyponatremia occurred. Hyponatremia was defined as the serum sodium ion concentration less than 135 mmol/L measured once during hospitalization, which was determined as hyponatremia.
- Model Establishment. Extract the multivariate logistic regression analysis results of the risk factors (age ≥ 60 years old, GCS score ≤ 12 points, combined with acute epidural hematoma or brain contusion, combined infection or high fever) established in the first part of the study as the moderately strong association. A logistic regression model (a classification model and a type of linear model) was established, and the regression coefficients of each risk factor were extracted as the score of each risk factor, and an early warning score table for craniocerebral injury complicated with hyponatremia was established.
- Efficacy Evaluation. Calculate the specific scores of the patients in the hyponatremia group and the normal serum sodium group according to the early warning score table. The scores are arranged in ascending order, and multiple different critical values are set between the lowest score and the highest score, draw the ROC curve, the larger the area under the ROC (receiver operator characteristic curve) curve, the better the energy efficiency [11].
- Risk Classification. Calculate the Youden index (the sum of sensitivity plus specificity minus 1) according to the sensitivity and specificity of each group. The larger the Youden index, the better the effect of the screening experiment and the greater the authenticity. Finding the score corresponding to the sensitivity and specificity when the Youden index is the largest, when it is less than this score, it is a low-risk group, and when it is greater than this score, it is a high-risk group. The medical information warning is shown in Figure 1.

(v) Monitoring of Vital Signs. The researchers communicated with doctors and responsible nurses and closely monitored the blood pressure, pulse, and respiration, especially the state of consciousness of patients in the high-risk group. Once it is found that the disturbance of consciousness is aggravated and clinical manifestations such as apathy, irritability, and lethargy appear, be alert to the occurrence of hyponatremia, and test serum sodium ions in time.

The sample size calculation formula when sampling survey is used and the analysis index is count data [12, 13]:

(5) $$\begin{array}{c} N=\frac{ZPQ}{d^{2}}, \end{array}$$

where *α* is the significance level, set at 0.05.

The Kendall harmony coefficient is calculated by SPSS 16.0 software, and the calculation formula is [14]

(6) $$\begin{array}{c} W=\frac{12}{m^{2}-\left(n^{2}-n\right)}\overset{n}{\underset{j=1}{\sum }}d_{j}^{2}. \end{array}$$

*n* represents the number of nursing-sensitive indicators, and *m* represents the total number of experts who have been consulted [15].

The formula for calculating the coefficient of variation is [16, 17]

(7) $$\begin{array}{c} \text{CV}=\frac{S}{x}. \end{array}$$

*S* is the standard deviation.

Infectious disease dynamics models for intra- and interhost coupling [18]:

(8) $$\begin{array}{c} \frac{ds}{dt}=A-\beta ES-\mu S,\\ \frac{dI}{dt}=\beta ES-\left(\mu +\sigma \right)S,\\ \frac{dE}{dt}=\theta IV\left(s\right)\left(1-E\right)-\gamma E. \end{array}$$

*E*(*t*) is the slow time term [19].

### 3.4. Comparison of Main Data of Traumatic First-Aid Deaths

According to the survey results of emergency death cases in 2018, four indicators of prehospital death were selected, including the fatality rate on arrival at the scene, the in-hospital response time of the ambulance, the time of the ambulance arriving at the scene, and the disposal rate of various prehospital first aid measures. Four indicators were compared, including the 1-minute attendance rate of the first-visiting doctor, the 5-minute attendance rate of second-line or superior doctors, the 30-minute attendance rate of consulting doctors, and the treatment rate of various emergency measures in the emergency department. Six indicators were compared, including in-hospital ward deaths selected for the first doctor's order issuance rate within 5 minutes, the consultation physician's attendance rate within 30 minutes, the start rate of blood transfusion within 30 minutes, the start rate within 30 minutes of surgery, the report rate of routine blood tests within 15 minutes, and the report rate of biochemical tests within 15 minutes. The ambulance rescue process is shown in Figure 2.

### 3.5. Influencing Factors of Prehospital Emergency Death

The age, gender, occupation, location of injury, time of injury, injury mechanism, method of arrival, whether or not to be transferred, time of admission, hospital level, place of death, and cause of death for patients with severe craniocerebral injury and fractures were selected as 12 factors that may affect emergency death as the research indicators, and quantify and assign values to the above variables. The names and assignments of the research factors are shown in Table 2.

### 3.6. Statistical Analysis

SPSS (Statistical Product Service Solutions), “Statistical Product and Service Solutions” software, was used. The original software was called “Statistical Package for Social Sciences.” The data were imported into SPSS 16.0 software, and the statistical methods included descriptive statistics, mean, standard deviation, *f* test, variance analysis, and multiple linear regression description. *P* < 0.05 was considered statistically significant difference.

The frequency table was made by counting the calling time, ambulance arrival time, age, gender, cause of injury, injury site, injury area, and PHI score (for example: a score of 0 to 3 is considered a minor injury; a score of 4 to 5 is considered a serious injury) of the patients with severe craniocerebral injury and fractures, and use Excel 2007 to calculate side-by-side charts to study the distribution law of trauma epidemiology [20].

(9) $$\begin{array}{c} \frac{dT}{dS}=\Lambda -KVT-MT,\\ {\left(\frac{dT}{DS}\right)}^{*}=KVT-\left(M+D\right)T,\\ {\left(\frac{dV}{DS}\right)}^{*}=PT-\text{CV}+g\left(E\left(t\right)\right). \end{array}$$

*DS* is the fast time item. The corresponding time variable is *S*.

It is assumed that any solution (*T*(*S*), *T*^∗^(*S*), *V*(*S*)) of the model satisfies the following initial conditions [21]:

(10) $$\begin{array}{c} T\left(S\right)>0,T^{*}\left(0\right)>0,V\left(0\right)>0. \end{array}$$

The basic reproduction number of virus infection in the host is defined as [22]

(11) $$\begin{array}{c} R_{W}=\frac{KPT}{C\left(m+d\right)}. \end{array}$$

When *g*(*E*) = 0, the model always has an infection-free equilibrium point.

(12) $$\begin{array}{c} T=\frac{c\left(m+d\right)}{kp},\\ T^{*}=\frac{cm}{kp}\left(R-1\right),\\ V=\frac{pmp}{c\left(m+d\right)}\left(1-\frac{1}{R}\right). \end{array}$$

Among them, *R*>1.

Considering the following scalar reaction-diffusion formula,

(13) $$\begin{array}{c} \frac{\partial }{\partial t}u\left(t,x\right)=D\Delta u\left(t,x\right)+\vartheta -\rho u\left(t,x\right), \end{array}$$

in which *u*, *ϑ*, *ρ* are normal numbers.

## 4. Results of Nursing Methods in Ambulances for Patients with Severe Traumatic Brain Injury and Fractures

Figure 3 shows the calculation accuracy according to the prehospital diagnosis and prehospital operation experimental data of the two groups, respectively. In the first group, the positive rate of prehospital diagnosis was 80.00%, the specific rate (the patient's own anticancer cells are cultured in vitro and then infused back into the patient's body to achieve the purpose of scientific anticancer) was 64.44%, the positive rate of prehospital operation was 82.22%, and the specific rate was 80.00%. The positive rate of prehospital diagnosis in the second group was 55.55%, the specific rate was 64.44%, the positive rate of prehospital operation was 64.44%, and the specific rate was 84.44%. It is believed that the positive rate of prehospital diagnosis and prehospital operation using the prehospital trauma assisted diagnosis and treatment system is higher than that of the onsite decision-making method, but the specific rate is lower.

The statistical results of the prehospital trauma assistant diagnosis and treatment system are shown in Table 3. It can be considered that the prehospital diagnosis of simulated craniocerebral trauma using the prehospital trauma assistant diagnosis and treatment system has a higher diagnostic positive rate than the onsite decision-making prehospital emergency, and the specificity is equivalent. Therefore, the system can better complete the prehospital diagnosis of craniocerebral trauma under simulated state.

The longest time for ambulances to arrive at the scene and to the hospital in each administrative area of the city is in area C, with a median of 11.03 and 29.68 minutes, respectively. The comparison of the time between the ambulance arrival at the scene and the arrival at the hospital is shown in Figure 4.

The distribution of injury causes in different age groups is shown in Table 4.

The distribution of injured sites in different age groups is shown in Figure 5.

Regarding the care factors of nonemergency transport services, the samples have the highest degree of care about formal legality and medical safety, and the average score is close to 5 points. Relatively speaking, relatives of patients with severe craniocerebral injury and fractures care less about service attitude or service price. The nonemergency transport services care about factors as shown in Table 5.

On the whole, the sample's overall evaluation of the hospital's nonemergency transport services is relatively low, with an average score of 7.11 points. On the whole, they showed high satisfaction with out-of-hospital nonemergency transport services, with an average score of 8.06. At the same time, for the level of medical care and ambulance equipment, they all showed a high satisfaction attitude, and the average score was higher than the overall evaluation score. Relatively speaking, the sample's satisfaction with the car-use process and the charging price is relatively low, with an average score of 8.02 and 6.59 points, which is lower than the overall evaluation of 8.06 points. However, the above analysis found that the sample cares the least about the charging price, and the sample as a whole shows a high evaluation of the nonemergency medical transfer service, indicating that the satisfaction of the lower charging price does not affect the overall satisfaction. Satisfaction with lower charged prices may simply be related to consumers' psychological expectations. The evaluation of transshipment services is shown in Table 6.

Nearly 70% of the respondents have used an ambulance only once, and only 6.8% have used it three or more times.  Figure 6 shows the ambulance use and basic attitude of relatives of patients with severe craniocerebral injury and fractures.

In terms of the purpose of using ambulances, 60% of the samples sought better treatment for transfer; 60% of the respondents learned the contact information of the transfer agency through the introduction of hospital staff. In addition, 40% of the relatives of patients with severe traumatic brain injury and fractures could not correctly judge the qualifications of the ambulance used. They mainly rely on body markings, medical staff's dress/professional level, and consultation with hospital staff to judge the qualifications and sources of the ambulances they use. The purpose of using an ambulance is shown in Figure 7.

The KMO (Kaiser-Meyer-Olkin) test statistic is an indicator used to compare simple and partial correlation coefficients between variables. For the nonemergency transport service, the KMO value was 0.801 > 0.7 in factor analysis, and it passed the Barth's sphericity test. And it can be seen from the above that the factor loading coefficient values corresponding to each item are all higher than 0.7, and the lowest is 0.740. Therefore, it shows that the nonemergency transport service evaluation data involved in this study has a high level of structural validity, and the research samples can be used for subsequent analysis and research. The construct validity test is shown in Figure 8.

Under the vast majority of indicators, the peak value of the good condition in the bar graph is decreasing, and the peak value of the aggravating condition is increasing, so it can be qualitatively explained that the treatment time in the emergency department is prolonged, and the overall condition is aggravated. The analysis of the risk degree of pulse beat is shown in Figure 9.

## 5. Discussion

The accident readiness intervention plan of clinical nurses developed based on accident rescue theory has applicability and has positive significance for improving the accident readiness of clinical nurses. Learning from the international advanced rescue experience, contacting the current clinical nurse training practice, comprehensive multimedia teaching materials and various teaching methods to actively carry out the theory, knowledge and skill training of accident nursing can promote the improvement of the accident rescue ability of local nurses.

The accident nursing teaching curriculum in China is relatively scattered, the nurses lack the opportunity to receive systematic accident nursing education, and the disaster relief skills and accident management ability are insufficient. In addition, in the implementation of accident rescue, Chinese clinical nurses still have insufficient accident rescue knowledge reserve, lack of core competence of accident nursing, low professional development ability of accident nursing, need to improve the level of knowledge, belief, and practice in response to accident events, and strong demand for accident nursing training. Cerebral salt wasting syndrome (CSWS) and syndrome of inappropriate secretion of antidiuretic hormone (SIADH) in patients with craniocerebral injury, in addition to the central nervous system damage caused by the disease itself, lead to a decrease in serum sodium ion concentration. Insufficient intake (such as fasting and eating disorders) or improper absorption (such as vomiting and diarrhea), use of dehydrating diuretics, etc. may also cause a decrease in serum sodium ion concentration. The two main causes of hyponatremia in patients with traumatic brain injury are cerebral salt wasting syndrome (CSWS) and syndrome of inappropriate secretion of antidiuretic hormone (SIADH). The pathogenesis of CSWS: central nervous system lesions or surgery, trauma, and other factors stimulate the hypothalamus and other parts, which can lead to increased secretion of atrial natriuretic peptide (ANP) and brain natriuretic peptide (BNP) and lead to increased glomerular filtration rate, increased salt and water excretion, and cerebral salt wasting syndrome (CSWS). After cerebral contusion and laceration, there will be ischemia and hypoxia in the brain tissue. The brain cells are directly damaged, and a large amount of calcium ions flow back into the cells, causing metabolic disorders of membrane phospholipids, reducing the generation of adenosine triphosphate and enhancing the lipid peroxidation reaction of brain cell membranes, which indirectly stimulate the hypothalamus, further triggering hyponatremia. Patients with craniocerebral injury have a large loss of sodium ions and insufficient intake due to disturbance of consciousness, nausea, vomiting, surgical trauma, use of dehydrating diuretics, and other reasons. Hyperthermia will make the loss of sodium ions more serious, and the risk of hyponatremia will also increase.

Healthy China is inseparable from medical support, but also needs the assistance of nursing. Nursing has gradually become a key force in promoting Healthy China. At present, the accident preparedness and emergency response ability of Chinese nurses still need to be improved. The domestic research on learning from the international advanced accident rescue experience is still limited, which shows that the research related to accident nursing in China has not yet been fully integrated with the international standards, and the theoretical guidance and disaster rescue skills need to be improved.

Accident readiness is one of the main indicators to measure the accident nursing ability of nurses. The level of accident readiness of clinical nurses and how to effectively improve the accident readiness of clinical nurses are still unclear. Therefore, on the basis of reviewing domestic and foreign researches on accident nursing and rescue, this study is based on the current situation of accident nursing and rescue in this region. Based on the accident rescue theory, the clinical nurses' accident preparedness intervention plan was developed, and the application effect of the intervention plan in the accident preparedness of clinical nurses in China was discussed by organizing and implementing relevant training, so as to provide a practical basis for the accident rescue training of clinical nurses, in order to further improve the quality of clinical nurse accident rescue.

Understanding the current level of nurses' accident readiness and analyzing the factors that affect nurses' accident readiness will help nursing managers to formulate strategies to improve nurses' accident readiness. In terms of disaster response skills, the multimedia teaching provided by Skype online teaching emphasizes that the curriculum setting of disaster response skills should be based on students' needs assessment, combining theory with practice. Early warning stage: nurses must master the characteristics of accident events, prepare disaster response resources and equipment, and respond to the evacuation system as soon as possible. Disaster classification phase: nursing students should use professional judgment to quickly classify casualties into categories such as immediate medical care, delayed care, nonurgent or minor, and fatal. First-aid knowledge and skills: nursing students should be proficient in rescue skills such as cardiopulmonary resuscitation, shock treatment, bleeding control, and splinting. Online teaching promotes the reflection and interaction of nursing students in their learning, practicing disaster relief skills through virtual disaster scenes, experiencing various rescue roles, and also improving teamwork and communication skills in postdisaster management. Online training, disaster drills, training drills, and interactive forums provided by Skype teaching mode are the most effective teaching methods. Nurses should master the knowledge and skills of postdisaster management through online courses, including ethical and moral principles, postdisaster psychological rehabilitation, advanced life support, disaster relief supplies, elimination of secondary injuries, and joint multiteam organization and collaborative management. Online courses based on Skype can ensure the relevance and timeliness of teaching content, help students to form their own knowledge system, and develop the accident management ability of nursing students.

Taking the theoretical knowledge and skills of accident rescue as the main training content, the training methods such as theoretical training, simulation teaching, and situational drills are integrated. Under the guidance of clinical nursing experts, the training outline, training materials, and training videos were compiled, and an accident readiness intervention plan suitable for Chinese clinical nurses was developed. It adopts a combination of training courses, centralized learning in departments, simulated onsite drills, and self-study. Among them, theoretical lectures mainly teach the theoretical construction, implementation methods, and medical system of accident rescue in Israel; special lectures teach the specific implementation rules and management of accident rescue. Multimedia teaching uses the combination of audiovisual and video to reproduce the disaster scene, which makes the rescue process more step-by-step and detailed and strengthens the training effect. Group discussion is to divide nurses into groups, set up relevant accident scenarios, and discuss according to their own accident rescue knowledge so that the theoretical knowledge of accident rescue can be effectively applied to specific cases.

Regardless of whether there is disaster relief experience, it has a significant positive effect on training, and the training effect of nurses without disaster relief experience is better than that of nurses with disaster relief experience. Nursing managers should strengthen accident rescue drills, help clinical nurses improve accident skills in practice, and set up different disaster rescue skill training courses according to the characteristics of nurses in different departments to ensure that nurses of different natures can effectively improve accident skills through different channels.

## 6. Conclusion

The accident preparation degree of nurses directly affects the quality of accident rescue. The results of the first part of this study also show that the training experience of clinical nurses is one of the main factors affecting their accident readiness. Nurses with sufficient accident knowledge can provide theoretical guidance for disaster rescue, and skilled disaster rescue skills are the key factors to ensure the quality of accident rescue. In addition, nurses' accident management ability is related to the smooth development of postdisaster reconstruction. Therefore, developing an accident readiness intervention program to improve the accident readiness of clinical nurses is essential to improve the quality of accident care. Learning from the international advanced rescue experience, contacting the current clinical nurse training practice, comprehensive multimedia teaching materials and various teaching methods to actively carry out the theory, and knowledge and skill training of accident nursing can promote the improvement of the accident rescue ability of local nurses. This study only retrospectively analyzed the medical records of patients with craniocerebral injury in one hospital. The sample size is small, and there may be selection bias; further large samples and multicenter cohort studies are needed to verify the results of this study. In the future work, systematic problems and countermeasures will be analyzed for each module of the ambulance medical emergency system, and the optimal allocation of prehospital medical resources and the optimal layout of emergency stations will be explored to improve the scientific feasibility of the research results.

## Figures and Tables

**Figure 1:** Medical information warning.

**Figure 2:** Ambulance rescue process.

**Figure 3:** Calculate the correct rate according to the experimental data of prehospital diagnosis and prehospital operation of craniocerebral trauma in the two groups, respectively.

**Figure 4:** Comparison of the time between the ambulance arriving at the scene and arriving at the hospital.

**Figure 5:** Distribution of injured sites in different age groups.

**Figure 6:** Ambulance usage and basic car usage attitude of relatives of patients with severe head injury and fractures.

**Figure 7:** Purpose of using an ambulance.

**Figure 8:** Construct validity test.

**Figure 9:** Analysis of the risk degree of pulse beating.

**Table 1:** Specific identification information.

Part	Cranial		
1	Open injury	Closed injury	Scalp avulsion
2	Periocular cyanosis, otorrhea, rhinorrhea, etc.	Otorrhea, rhinorrhea, malformation, localized hematoma, etc.	Otorrhea, rhinorrhea, fluctuating hematoma, etc.
3	Urinary incontinence, fecal incontinence, foreign body incontinence, etc.	Severe pain, etc.	Delirium, epilepsy, etc.
4	Negative meningeal irritation sign GCS score	Negative meningeal irritation sign GCS score	Negative meningeal irritation sign GCS score

**Table 2:** Study factor names and assignments.

Factor name	Assign
Arrival method	1, arrival by ambulance; 2, arrival by nonambulance
Whether to transfer	1, transfer from another hospital; 2, nontransfer
Admission time	1, day; 2, last night; 3, next night
Hospital grade	1, nontertiary hospital; 0, tertiary hospital
Place of death	1, emergency department; 0, hospital ward
Cause of death	1, nontraumatic brain injury; 0, traumatic brain injury

**Table 3:** Statistical results of prehospital trauma assistant diagnosis and treatment system.

Relevant factors		On-the-spot decision		Total
		Positive	Negative	
Prehospital trauma assistant diagnosis and treatment system	Positive	20	16	36
	Negative	5	4	9
Total		25	20	45

**Table 4:** Distribution of injury causes in different age groups.

Type of injury	0–22		23–35	
	Number of people	Composition ratio (%)	Number of people	Composition ratio (%)
Glass scratches	6	1.69	659	0.5
Traffic injury	30	42.02	25575	36.59
Brawl injury	1112	24.65	16562	14.34
Stab wound	9	823	3180	1.86
Fall from height	1484	3.16	1863	2.26

**Table 5:** Nonemergency transport services care about factors.

Care factor	Highest score	Lowest score	The average score	Standard deviation
Ease of use	1.00	6.00	3.22	1.37
Timeliness	1.00	6.00	3.15	1.19
Service attitude	1.00	6.00	2.70	1.17
Service fee	1.00	5.00	1.82	1.16

**Table 6:** Evaluation of transshipment services.

Evaluation item	Average value	Standard deviation
Out-of-hospital nonemergency transfer medical service level	8.45	1.80
Out-of-hospital nonemergency transport ambulance equipment	8.80	1.48
Out-of-hospital nonemergency transfer to a vehicle	8.02	1.79
Out-of-hospital nonemergency transfer charges	6.59	2.31
Overall evaluation of out-of-hospital nonemergency transport services	8.06	1.58
Overall evaluation of hospital nonemergency transport services	7.11	2.19

## Data Availability

No data were used to support this study.
